The article "Clinical Treatment and Nursing Intervention Study of Clipping Treatment of Cerebral Aneurysm under the Health Model of Data Analysis" was retracted in 2023. Reasons: signs of a paper mill; suspected computer-generated content; unreliable results or conclusions; lack of ethics approval or compliance.

# Clinical Treatment and Nursing Intervention Study of Clipping Treatment of Cerebral Aneurysm under the Health Model of Data Analysis

**DOI:** 10.1155/2022/8178963

**Published:** 2022-06-30

**Authors:** Yuyou Huang, Liping Huang

**Affiliations:** Emergency Intensive Care Unit, Longhua People's Hospital, Shenzhen 518000, Guangdong, China

## Abstract

Middle cerebral artery aneurysm is a common type of intracranial aneurysm in neurosurgery, accounting for about 20% of intracranial aneurysms, and is the third most common site of intracranial aneurysms. The surgical success rate and postoperative recovery ability of today's treatment plans are not satisfactory. Therefore, this paper designs a health model based on data analysis to clinically apply clipping surgery for cerebral aneurysm. This paper studies data analytics health models in the context of big data analytics. The model combines the characteristics of cerebral aneurysms for targeted analysis, and then through the understanding of the clipping treatment of cerebral aneurysms, this paper combines the deep learning in the neural network to train the treatment plan under the data analysis health model. Finally, this paper designs a therapeutic plan for clipping treatment of cerebral aneurysm based on a data analysis health model. To verify its data analysis ability, this paper designs experiments on unbalanced data sets and experiments to improve the execution efficiency of the algorithm. After analyzing the results obtained from the experiment, this paper will apply them to the clinic. The final experiment showed that the surgical success rate of the clipping treatment for cerebral aneurysm based on the data analysis health model was increased by 21.84% compared with the traditional clipping treatment for cerebral aneurysm.

## 1. Introduction

With the advent of the era of big data, medical informatization has had a huge impact on the domestic medical industry and promoted the advancement and reform of the entire industry. Medical information is based on various basic medical data such as clinical and monitoring data collected directly from hospitals, research data from medical research institutions, and personal health data collected directly by individuals.

Brain aneurysms can be divided into three types: aortic aneurysm, branch aneurysm, and distal aneurysm according to the location of growth, usually at the origin of the anterior cranial artery. The neck of the tumor is generally wide and closely associated with perforated blood vessels. The risk of postoperative brain aneurysms is much higher than elsewhere. Branch aneurysms have the highest incidence, about 80–85%, usually in the initial branch of the middle cerebral artery, mainly in cerebral aneurysms or giant aneurysms. Distal aneurysms are mainly caused by infectious factors, which are rare in clinical diagnosis and treatment. If data analysis can be applied to a healthy model to improve the clipping treatment of cerebral aneurysms and optimize its postoperative care, it can improve the surgical success rate and postoperative recovery of patients with cerebral aneurysms.

The article "Clinical Treatment and Nursing Intervention Study of Clipping Treatment of Cerebral Aneurysm under the Health Model of Data Analysis" was retracted in 2023. Reasons: signs of a paper mill; suspected computer-generated content; unreliable results or conclusions; lack of ethics approval or compliance.

The innovation of this paper is that this paper combines the health data analysis model of big data and then analyzes the surgical plan for the clipping treatment of the cerebral aneurysm. Then, through the application of deep learning of neural network in data analysis health model, a treatment plan for clipping treatment of cerebral aneurysm based on big data analysis health model is finally designed. This paper designs experiments on unbalanced data sets and experiments to improve the execution efficiency of the algorithm, and tests and improves the performance of the data analysis model.

## 2. Related Work

Mobile devices are increasingly becoming an integral part of people's daily lives, facilitating a variety of useful tasks. Tawalbeh LA describes a cloudlet-based mobile cloud computing infrastructure for healthcare big data applications. He reviews the techniques, tools, and applications of big data analytics and concludes the design of networked healthcare systems using big data and mobile cloud computing technologies [1]. He applied big data to the medical system. If he can design a data analysis health model, it will be more useful for this article. To explore the risk factors and intervention strategies of cerebral arteriovenous malformation complicated with aneurysm hemorrhage, Li X collected and analyzed the clinical and imaging data of 42 cases of cerebral arteriovenous malformation complicated with aneurysm [2]. According to the results of intraoperative angiography and the characteristics of vascular structure, the treatment plan is formulated. Brain aneurysm rupture is closely related to aneurysm size. Because aneurysms often have complex shapes, using only the size of the aneurysm dome and neck may be inaccurate, and important geometric information may be overlooked. Dong B proposed a level-set-based surface capture algorithm to first capture aneurysms from the vessel tree [3]. Since aneurysms are described by level-set functions, the volume, curvature, and other geometric quantities of the aneurysm surface can be easily calculated for medical research. The purpose of Byndiu AV is to study the characteristics of early clinical neurological manifestations after intraoperative rupture of an aneurysm (AA) [4]. He then conducted a retrospective study of the surgical outcomes of 69 patients with hemorrhagic acute cerebrovascular disease due to ruptured cerebral aneurysms, including intraoperative ruptures. The increasing popularity and development of data mining technology have brought a serious threat to the security of sensitive personal information. Xu L takes a broader perspective on privacy issues related to data mining and studies various methods that help protect sensitive information [5]. He identified four different types of users involved in data mining applications, namely data providers, data collectors, data miners, and decision-makers. Machine learning prediction methods are highly effective in applications ranging from medicine to assigning city fire and sanitation inspectors. Thus, Athey S's research is mainly focused on making predictions and making decisions and requires an understanding of the underlying assumptions to optimize data-driven decision-making [6]. Advances in information technology have witnessed tremendous advancements in healthcare technology in various fields today. However, these new technologies have also made healthcare data not only larger but more difficult to process. To provide a more convenient healthcare service and environment, Zhang Y proposed a cyber-physical system for patient-centric healthcare applications and services based on cloud and big data analysis technology, called Health-CPS [7]. To sum up, most of the cited literature is about big data and cerebral aneurysms. If the data analysis of big data can be applied to the health model, and then analyzed for clipping treatment of cerebral aneurysms, it will be more in line with the theme of the article. Therefore, it is necessary to further study the application of data analysis of big data in health models.

The article "Clinical Treatment and Nursing Intervention Study of Clipping Treatment of Cerebral Aneurysm under the Health Model of Data Analysis" was retracted in 2023. Reasons: signs of a paper mill; suspected computer-generated content; unreliable results or conclusions; lack of ethics approval or compliance.

## 3. Design Method of Health Model Based on Big Data

### 3.1. Big Data Analysis Model

#### 3.1.1. Big Data

In recent years, with the rapid development of the Internet society, a large amount of information has been digitized, and big data [8] has emerged as the times require. Modern people are all surrounded by this massive amount of data. The most notable feature of big data is its huge amount of data. Common computer storage units of measurement have developed from GB to TB, PB, EB, ZB, YB, etc. Taking the world's largest search engine Google as an example, its daily data processing volume has exceeded 24 PB, which is already equivalent to 2 to the 50th power of bytes, and a 4 MB ordinary MP3 song can be played for 48,000 years. The fields involved are shown in Figure 1.

#### 3.1.2. Characteristics of Big Data

Big data involves a huge amount of data with a wide variety of types. It is necessary to use software to complete the processing of relevant data sets within a certain period and analyze the basis for decision-making references to reflect the value of big data. Big data has the following characteristics:

1. The amount of data is huge and complex [9], and the amount of data is huge. In general, traditional databases do not have the function of collecting and saving, and there are various types of data, which come from various aspects, and the sources are extremely complex, presenting various structures and various media forms, which far exceed the previous database capabilities. To realize the role of big data technology in promoting economic development, management and analysis need a database with powerful functions, which can lead to the potential value of data [10].
2. The processing speed is fast [11]. Big data has higher and higher requirements for computer technology, and data will change in various ways, so it is particularly important to process data on time. In addition to data collection, data analysis and mining are required [12]. Therefore, to meet real-time reference requirements, data must be analyzed and processed rapidly and continuously.
3. It uses data analysis to obtain valuable information [13]. The core of big data is not the storage and simple processing of huge amounts of data, but the specific analysis of these data, and then draw some important information from it. For example, after analyzing the shopping lists of a large number of customers, a supermarket found that beer often appeared on the same shopping list as diapers. The supermarket concluded that customers who buy beer usually also buy diapers, so they put beer and diapers together on the product placement, which not only makes it easier for customers to get the product but also increases the sales of these two products. In the above case, the supermarket has obtained valuable information for its operation through the analysis of the data. The same is true for big data technology, but the amount of data is larger, and the processing and analysis methods are more complicated.

#### 3.1.3. The Basic Value of Big Data

Today, big data has become a key element in transforming production relations and improving social productivity. When it comes to the value of big data, we cannot avoid considering the huge economic benefits contained in it from the perspective of social attributes. The concept of “data is an asset” is particularly important in the era of big data. The industrial chain derived from the element of “data” covers data itself, technology, and thinking.

From the perspective of big data itself, the possession of massive data by an enterprise is equivalent to obtaining a “rich mine” of future competition, which is tantamount to controlling a large number of production materials and winning the ownership of data [14]. Big data owners can not only use big data resources but also make secondary use of data, improve user experience, and improve their operations and services [15]. It is also possible to transfer the use value of massive data to third-party technology companies through data authorization, so as to obtain its value and improve economic benefits. It is foreseeable that a large number of such “data middlemen” will emerge shortly, such as banks, search engines, e-commerce platforms, social industries, government departments, and so on. Mastering big data itself occupies the core position of the big data industry chain. Taking the gold mine as an analogy, whether it is its miner or its seller, the owner who benefits the most is ultimately its owner.

The article "Clinical Treatment and Nursing Intervention Study of Clipping Treatment of Cerebral Aneurysm under the Health Model of Data Analysis" was retracted in 2023. Reasons: signs of a paper mill; suspected computer-generated content; unreliable results or conclusions; lack of ethics approval or compliance.

From the perspective of big data skills, in the early days of the big data era, only those who take the lead in mastering advanced data processing methods can capture the greatest commercial value. What has to be mentioned here is a big data technology and big data talents. Big data technology is to “make data sound” through technical means, that is, to develop the potential value and innovative uses of data from the vast ocean of data. Undoubtedly, the monopoly of related technologies in data mining, data analysis, and data presentation in the future will be enough to make consulting service companies, technology suppliers, and information analysis companies become industry leaders. At the same time, big data talents will also gain a pivotal position. Today, conclusions based on technical and data facts are far more convincing than those guided by traditional experience, and data scientists will replace industry experts as the dominant force in future strategic decisions.

From the perspective of big data thinking, the value of big data lies in the emancipation of the mind, that is, to get rid of the influence of inherent patterns and vested interests, and to “dissect sparrows” from the height of top-level design. From a methodological point of view, it is to jump out of the shackles of thinking in the era of small data and use quantitative thinking, overall thinking, relevant thinking, and fault-tolerant thinking in the era of big data to guide people to understand and transform the world from a new perspective.

#### 3.1.4. Application of Big Data

The arrival of the era of big data has affected all aspects of social development in all countries in the world, from business and economics to healthcare, technology, education, and more. As long as it is closely related to people's lives, big data is everywhere [16]. Therefore, whether it is the rise and development of the big data industry or as a technical means, big data has been widely used in various fields. Therefore, the application of big data mentioned here is not only the application of big data technology in other fields but also the positive impact of the integration of the big data industry in other industries.

The article "Clinical Treatment and Nursing Intervention Study of Clipping Treatment of Cerebral Aneurysm under the Health Model of Data Analysis" was retracted in 2023. Reasons: signs of a paper mill; suspected computer-generated content; unreliable results or conclusions; lack of ethics approval or compliance.

Big data is a strategic resource that is vigorously developed in China, mainly because big data can be extended to various fields as a technology. After the Internet of Things and cloud computing [17], the development and application of big data technology have received attention from all walks of life. The biggest achievement of big data applications is their integration. It is not only the integration and development of related industries but also integration with industrial clusters. Only in the process of integration and application can big data play its role. The subdivision of its application can be summarized into three aspects, the application of data storage; the application of data analysis; and the application of data fusion. It is the application of these three aspects that allows big data to penetrate all aspects of other industries, and even more subtle links.

#### 3.1.5. Research on Health Big Data

Health big data [18, 19] refers to all data closely related to human health and public health, including birth, infant health management, vaccination, admission inspection, employment inspection, medical treatment, hospitalization, exercise, sleep, death, and other life cycles. It can be roughly divided into structured data such as inspection data and semi-structured and unstructured data such as medical record data and medical images. Test data mainly refer to data generated by routine blood tests, cell tests, and pathological tests of various organs. Medical record data refers to data related to personal medical diagnosis information records and health status, etc., which are usually managed electronically. Medical image data refer to images such as internal tissue structures obtained from the human body. Through this part of the data, a more detailed understanding of the health status of the human body can be obtained.

The rapid development of information technology and social changes have gradually transformed traditional medical and health records from paper files to digital storage and gradually entered the era of big data in the medical industry. The development process of China's healthcare informatization is shown in Figure 2.

Health big data has the characteristics of redundancy, polymorphism, privacy, timeliness, and incompleteness, so the analysis and processing of health big data is a new challenge. Common methods for data analysis of health big data include feature analysis, classification, regression analysis, clustering, and visualization. Combining machine learning technology to reason and judge different types of test data, medical record data, medical images, and other data is a new means to strengthen medical services, predict disease conditions and reduce medical costs.

The article "Clinical Treatment and Nursing Intervention Study of Clipping Treatment of Cerebral Aneurysm under the Health Model of Data Analysis" was retracted in 2023. Reasons: signs of a paper mill; suspected computer-generated content; unreliable results or conclusions; lack of ethics approval or compliance.

#### 3.1.6. Traditional Algorithm of Health Big Data

Classification is to use the known attribute data of the data set [20] to infer an unknown discrete attribute data. The key to making accurate predictions is to establish an effective model between known attribute information and unknown discrete attributes, that is, a classification model. Therefore, the classification problem includes two processes of learning and classification, as shown in Figure 3.

Traditional health data classification methods [21] are mainly based on supervised learning. In machine learning, common classification algorithms include SVM [22], decision tree [23], and so on. The classification of health data is actually to map the patient's inspection information to specific categories, so as to achieve the right medicine and accurate treatment.

When traditional supervised learning algorithms classify different types of healthy big data, preprocessing and feature selection are performed first, and then the classifier is trained. The conventional classification process of health big data is shown in Figure 4.

### 3.2. Clipping Therapy for Cerebral Aneurysms

Patients with cerebral aneurysms [24, 25] are often accompanied by intracranial hematomas. In the case of an intracranial hematoma, coma, or worsening of state after a brief hemorrhage, mainly due to cerebral vasospasm, not hematoma compression or brain herniation. Therefore, in patients with middle cerebral aneurysms and large intracranial hematomas, early aneurysm debridement and intracranial hematoma removal are recommended to prevent secondary rupture of the aneurysm.

Due to the special anatomical location and complex structure of MCA, most aneurysms have wide or irregular heads, and intracranial hematomas are easily formed after rupture, so they are not suitable for endovascular interventional therapy.

The release of ISAT in 2002 indicated that endovascular therapy is safer and more effective than surgical clipping. More and more clinicians use endovascular therapy to treat intracranial aneurysms, but ISAT results are clinical results 12 months after treatment. Although the study was for ruptured intracranial aneurysms, its publication also has major implications for how unruptured aneurysms are treated. Although in recent years ISAT showed that the difference between the two treatments decreased with the extension of follow-up time, the latest ISAT showed no significant difference between the two treatments. And only 303 of the 2143 patients in ISAT were MCAA, and middle cerebral aneurysms were underrepresented, but the endovascular treatment of intracranial aneurysms has become an important treatment method for aneurysms. There is no consensus on which of the two approaches provides long-term security. Although the location of the middle cerebral aneurysm makes it more likely that craniotomy clipping is a straightforward, feasible approach, there is both early vasospasm and additional damage from the craniotomy (for example, traction injury of brain tissue and perioperative hematoma). These difficulties and complications can be avoided with interventional therapy. However, there is no high-level, high-quality evidence that its therapeutic efficacy and safety are superior to craniotomy clipping.

The article "Clinical Treatment and Nursing Intervention Study of Clipping Treatment of Cerebral Aneurysm under the Health Model of Data Analysis" was retracted in 2023. Reasons: signs of a paper mill; suspected computer-generated content; unreliable results or conclusions; lack of ethics approval or compliance.

The specific operation process of craniotomy clipping treatment is as follows:

The main surgical instruments include microscopes and microscopic instruments, various types of aneurysm clips, and bipolar coagulation.

With the patient supine, the head is rotated 30 degrees in the opposite direction so that the zygomatic protrusion reaches the highest point of the surgical site. Due to the shallow position of the middle cerebral artery, during the craniotomy, the periosteum of the skull, lateral head muscle, and skull is squeezed from the subperiosteal to the front and lower parts, which shortens the time of the craniotomy. This prevents damage to the craniotomy, including the anterior branches of the facial nerve and the supraorbital nerve. In the internal carotid cistern, the bone hole on the junction of the coronary artery and the upper head line was pulled out, the flap was opened with a grinding knife, the sericoid bulge was removed, and the meninges were suspended, and the dura was cut into an arc. The sericin fissure was isolated under a microscope while opening to release cerebrospinal fluid to reduce intracranial pressure, and the middle cerebral artery was explored retrogradely along the internal carotid artery. Rupturing or hemorrhage may occur during dissection, and temporary clips are recommended to temporarily block the proximal parent artery, usually within 15 minutes. Choosing the appropriate aneurysm clip based on the size and orientation of the aneurysm neck. In the case of a large aneurysm, blood flow may be temporarily cut off. When the aneurysm sac remains, multiple clips can be used for clipping. Since the aneurysm is so large that complete clamping of one or more aneurysms is expected to be difficult, the aneurysm can be cauterized around the head of the aneurysm by bipolar low-frequency conduction, thus allowing the tumor to be clipped before resection. The temporary occlusion clip was released, and intraoperative fluoroscopy revealed that the parent artery was not occluded and no aneurysm was found. Bleeding was completely stopped before surgery, and the decision to replace the bone flap was based on intracranial pressure. Dehydration and decreased intracranial pressure, prophylaxis of vasospasm, hemostasis, anti-infectives, and other symptomatic and supportive treatments are routinely performed after surgery.

The article "Clinical Treatment and Nursing Intervention Study of Clipping Treatment of Cerebral Aneurysm under the Health Model of Data Analysis" was retracted in 2023. Reasons: signs of a paper mill; suspected computer-generated content; unreliable results or conclusions; lack of ethics approval or compliance.

### 3.3. Principles and Models of Neural Networks

Assuming that there is a training sample set, (*a*^(*i*)^, *b*^(*i*)^), taking the supervised learning neural network as an example, a high-order complex nonlinear hypothesis model *g*_*W*,*y*_(*a*, *b*) is constructed by using the neural network algorithm, and the parameters *W* and *y* are the parameters of the function. As shown in Figure 5, the general complex neural network model is described first from the simplest single neuron consisting of only one “neuron”.

In Figure 5, *a*_*k*_, (*k*=1,2,3…) is the input vector and *wk*, (*k*=1,2,3…) is the weight of each input component. The function of the weight can be regarded as the connection strength of each component, and the input component can be enlarged or reduced by changing the size of the weight. *d* is the excitation function, also known as the activation function, the transfer function. The *y* value is an offset value, also called a threshold.

When using data sets *a*_1_, *a*_2_, *a*_3_ as the input of the neuron model to train the network parameters, it is necessary to add a bias + 1 to it, and then use it as the input data of the neuron. Its output is expressed as

(1) $$\begin{array}{c} g_{w,y}\left(a\right)=g\left(W^{T}a\right)=d\left(\sum_{i=1}^{3}W_{i}a_{i}+y\right). \end{array}$$

Among them, the function *d*(*·*) is an activation function, and there are many choices, and specific choices are made according to different data objects. In general, the sigmoid function is used as the activation function *d*(*·*) in the neural network

(2) $$\begin{array}{c} d\left(c\right)=\frac{1}{1+\text{exp}\left(-c\right)}. \end{array}$$

In addition to the sigmoid function, the hyperbolic tangent function tanh, ReLu (Rectified Linear Units), etc., can be selected, and different activation functions can be selected according to the specific application background.

(3) $$\begin{array}{c} d\left(c\right)=\text{tan}g\left(c\right)=\frac{q^{c}-q^{-c}}{q^{c}+q^{-c}},\\ d\left(c\right)=\text{max}\left(0,c\right). \end{array}$$

As shown in Figure 6, layer1 is the input layer of the network, layer3 is the output layer of the network, and the middle layer layer2 is the hidden layer. Respectively, adding a bias unit in addition to the output layer:

In the specific calculation, it is necessary to transpose the original feature matrix, so that the features of the same data object are all in the same row of the training matrix and then use matrix multiplication to calculate, namely

(4) $$\begin{array}{c} c^{\left(2\right)}=\theta^{\left(l\right)}A^{T},\\ x^{\left(2\right)}=h\left(c^{\left(2\right)}\right). \end{array}$$

Since the *g*_*θ*(*a*)_ calculated by the forward propagation algorithm cannot obtain the best feature representation, it is also necessary to adjust the weights of the network to obtain the best network model.

The article "Clinical Treatment and Nursing Intervention Study of Clipping Treatment of Cerebral Aneurysm under the Health Model of Data Analysis" was retracted in 2023. Reasons: signs of a paper mill; suspected computer-generated content; unreliable results or conclusions; lack of ethics approval or compliance.

Here, it is necessary to optimize the network model by calculating the partial derivative (*∂*/*∂θ*_*ij*_^(*l*)^)*J*(*θ*) of the cost function *J*(*θ*) through the back-propagation algorithm, starting from the last layer of the network, and adjusting the weights of the network in reverse.

If the neural network model is a four-layer network training model, with (*A*(1), *B*(1)) as the training set of the network, the forward propagation algorithm is briefly described as:

(5) $$\begin{array}{c} x^{\left(1\right)}=a,\\ c^{\left(2\right)}=\theta^{\left(1\right)}x^{\left(l\right)},\\ x^{\left(2\right)}=h\left(c^{\left(2\right)}\right)\left(\text{add}x_{0}^{\left(2\right)}\right),\\ c^{\left(3\right)}=\theta^{\left(2\right)}x^{\left(2\right)},\\ x^{\left(3\right)}=h\left(c^{\left(3\right)}\right)\left(\text{add}x_{0}^{\left(3\right)}\right),\\ c^{\left(4\right)}=\theta^{\left(3\right)}x^{\left(3\right)},\\ x^{\left(4\right)}=h_{\theta }\left(a\right)=h\left(c^{\left(4\right)}\right). \end{array}$$

When the forward propagation is calculated, the back-propagation can be started based on the idea of the error (the deviation between the output value *x*^(4)^ and the actual value *b*(*n*) of the training set). The specific steps are as follows:

Taking the variable *δ* to represent the error, then

(6) $$\begin{array}{c} \delta^{\left(4\right)}=x^{\left(4\right)}-b. \end{array}$$

Using formula (9) to calculate the error of the previous layer

(7) $$\begin{array}{c} \delta^{\left(3\right)}={\left(\theta^{\left(3\right)}\right)}^{T}\delta^{\left(4\right)}*h^{\prime }\left(c^{\left(3\right)}\right), \end{array}$$

where *h*′(*c*^(3)^) is the derivative of the S-function.

(8) $$\begin{array}{c} h\prime \left(c^{\left(3\right)}\right)=x^{\left(3\right)}*\left(1-x^{\left(3\right)}\right). \end{array}$$

Then continue to calculate the error of the next layer

(9) $$\begin{array}{c} \delta^{\left(2\right)}={\left(\theta^{\left(2\right)}\right)}^{T}\delta^{\left(3\right)}*h\prime \left(c^{\left(2\right)}\right). \end{array}$$

Because the input layer of the network uses raw data as input, its error is 0. Finally, calculate the partial derivative (*∂*/*∂θ*_*ij*_^(*l*)^)*J*(*θ*) of the cost function

(10) $$\begin{array}{c} \frac{\partial }{\partial \theta_{ij}^{\left(l\right)}}J\left(\theta \right)=x_{j}^{l}\delta_{j}^{l+1}. \end{array}$$

The meanings of the superscript and subscript in the above formula: *l* represents the currently calculated network layer, and *j* represents the subscript value of the activation unit of the current calculation layer. This is also the next layer of additional characters for the *j*th input variable. *i* is represented as an additional character for neural network errors.

The article "Clinical Treatment and Nursing Intervention Study of Clipping Treatment of Cerebral Aneurysm under the Health Model of Data Analysis" was retracted in 2023. Reasons: signs of a paper mill; suspected computer-generated content; unreliable results or conclusions; lack of ethics approval or compliance.

When Δ_*ij*_^(*l*)^ is calculated, the error representation of the cost function can be expressed as:

(11) $$\begin{array}{c} D_{ij}^{\left(l\right)}=\frac{1}{m}\Delta_{ij}^{\left(l\right)}+\lambda \theta_{ij}^{\left(l\right)}\text{ if}j\neq 0,\\ D_{ij}^{\left(l\right)}=\frac{1}{m}\Delta_{ij}^{\left(l\right)}\text{ if}j=0. \end{array}$$

## 4. Data Analysis Model Performance Test Experiment

### 4.1. Experiments with Unbalanced Data Sets

In three groups of class-imbalanced purely numeric data sets, the traditional SMOTE algorithm and the improved SMOTE algorithm based on the centroid were used to balance the data sets and use random forests to predict the classification. By comparing the two results, the effect of the improved SMOTE algorithm can be verified. The information of these three sets of data sets is described in detail in Table 1:

As can be seen from Table 1, since the imbalance rates of these three data sets are all low, it is difficult to use the random forest to classify and predict the sample data set if there are few samples from the minority class. Therefore, both the traditional SMOTE algorithm and the modified gravity-based SMOTE algorithm are used to improve the imbalance of the data set. The data set will then be classified and predicted according to the random forest. Then, the experimental results are compared and analyzed using classification accuracy, ROC curve (AUC field), and F1-measure evaluation metrics.

From Tables 2–4, it can be seen that.

1. Due to the low imbalance rate of these three data sets, that is, due to the low proportion of the minority class in the entire data sample. Therefore, when using the random forest algorithm to directly classify these three data sets, although the classification effects of different data sets will change, it can be seen that the overall classification performance is not high.
2. Using the traditional SMOTE algorithm to synthesize a small number of samples, after improving the imbalance rate of the data set, use the random forest algorithm to classify and predict the data set. The classification performance on the three data sets has improved by an average of 10%. The results show that when the random forest algorithm is used to classify the data set, the imbalance of the data will have a certain impact on the classification results.
3. Balancing the data set using the improved SMOTE algorithm and then using the random forest algorithm to classify and predict the data set. By using the traditional SMOTE algorithm, the classification performance of the three sets of data is further improved, with an average increase of 3–5%. This result shows that the quality of the new samples synthesized by the improved SMOTE algorithm is very good.

The article "Clinical Treatment and Nursing Intervention Study of Clipping Treatment of Cerebral Aneurysm under the Health Model of Data Analysis" was retracted in 2023. Reasons: signs of a paper mill; suspected computer-generated content; unreliable results or conclusions; lack of ethics approval or compliance.

The original data set is balanced and transformed using the traditional SMOTE algorithm and the improved SMOTE algorithm. The experimental comparison results are shown in Figure 7.

Obviously, the average classification accuracy of the improved SMOTE algorithm is 4% higher than that of the traditional SMOTE algorithm, and the classification accuracy of the original data set without SMOTE algorithm is much lower. If the original data set is improved with the improved SMOTE algorithm, the AUC area will reach a maximum of 0.88, which is 0.04 higher than the traditional SMOTE algorithm, but the AUC area is only 0.72, using random forest to classify the original data set, but the classification performance is poor. This shows that using the traditional SMOTE algorithm to improve the imbalanced data set can improve the random forest classification performance. At the same time, the new samples synthesized by the improved SMOTE algorithm are of higher quality than the traditional SMOTE algorithm, and the classification effect of random forest is better.

### 4.2. Experiments to Improve the Efficiency of Algorithm Execution

To further demonstrate the impact of the improved algorithm in detecting global outliers, this paper uses a classification model to test the data sets processed by two different algorithms on the cerebral aneurysm test data set and analyzes and compares them through experiments. As in the supervised algorithm experiment, the labeled data in the data set are divided into two parts, one part is training data and the other part is test data, and the training data account for 70%. The difference is that the training data in the semi-supervised algorithm are also divided into two categories, one part is labeled data and the other part is unlabeled data. This division enables three different types of algorithms (supervised, unsupervised, and semi-supervised) to be trained and tested on the same data set, thereby improving the performance of the algorithms based on the performance analysis of different algorithms. The trained model is verified using the test set, and the experimental results obtained are shown in Table 5:

The outlier alignment before and after improvement, and the AUC change are shown in Figure 8.

The article "Clinical Treatment and Nursing Intervention Study of Clipping Treatment of Cerebral Aneurysm under the Health Model of Data Analysis" was retracted in 2023. Reasons: signs of a paper mill; suspected computer-generated content; unreliable results or conclusions; lack of ethics approval or compliance.

It can be seen from Figure 8 that the increase in the data set size also brings more outliers, and the improved algorithm can identify outliers more comprehensively than the original algorithm. The analysis shows that the improved algorithm further improves the performance of subsequent data analysis. Overall, the improved algorithm is better than the original algorithm in terms of execution time and detection of outliers. Among them, the reduction of the algorithm execution time becomes more and more obvious with the increase of the data set, and the performance of the classification model has also been improved to varying degrees.

## 5. Results of Cerebral Aneurysm Clipping Treatment

### 5.1. Tumor Observation and Analysis

The current gold standard for the diagnosis of intracranial aneurysm is whole-brain angiography. In this study, the image data selected for constructing the 3D model of the intracranial aneurysm were head CTA image data. To verify whether DSA and CTA measurement results were statistically different, the imaging data (data acquisition is performed under the same field of view, and the long and short diameters of the aneurysm body and the width of the aneurysm neck are measured, respectively, of 50 patients with intracranial aneurysms confirmed by head CT angiography and whole cerebral angiography were collected. SPSS 17.0 statistical software was used for data analysis and processing, and *P* < 0.05 was considered statistically significant. The experimental results are shown in Figure 9.

The measured values of the longest diameter, shortest diameter, and aneurysm neck width on 3D-CTA and 3D-DSA obeyed normal distribution. There was no significant difference in the mean value of aneurysm (long diameter, short diameter, and width) measured between the two groups (*P* < 0.05).

### 5.2. Control Experiments

The data collected through the experiment optimize the clipping treatment of cerebral aneurysm based on the data analysis healthy model designed in this paper. To explore the clinical treatment effect and postoperative nursing effect of this treatment plan, a set of controlled experiments were designed in this paper. The experiment was divided into two groups, one group used the clipping treatment plan for cerebral aneurysm based on the data analysis healthy model designed in this paper and the other group adopted the traditional clipping treatment plan for cerebral aneurysm. The success rate of surgery and the degree of postoperative recovery are shown in Figure 10.

The article "Clinical Treatment and Nursing Intervention Study of Clipping Treatment of Cerebral Aneurysm under the Health Model of Data Analysis" was retracted in 2023. Reasons: signs of a paper mill; suspected computer-generated content; unreliable results or conclusions; lack of ethics approval or compliance.

As can be seen from Figure 10, the surgical success rate of the clipping treatment for cerebral aneurysm based on the data analysis healthy model reached 92.93%. The traditional clipping treatment for cerebral aneurysm has a surgical success rate of only 71.09%. In contrast, the clipping treatment plan for cerebral aneurysm based on the data analysis health model designed in this paper has a 21.84% higher surgical success rate than the traditional clipping treatment plan for cerebral aneurysms. In contrast, the degree of postoperative recovery of the clipping therapy for cerebral aneurysm based on the data analysis healthy model recovered from 72.31% to 93.62% in the 5-month recovery period. The degree of postoperative recovery of the conventional clipping regimen for cerebral aneurysms only recovered from 65.41% to 73.41% in the 5-month recovery period. In summary, the surgical success rate and postoperative recovery ability of the clipping treatment plan for cerebral aneurysm based on the data analysis health model designed in this paper have been greatly improved.

## 6. Conclusions

This paper mainly studies the treatment plan and clinical care of clipping surgery for cerebral aneurysm based on a data analysis health model. Therefore, this paper formulates a health model based on the data analysis in big data and the content of cerebral aneurysm and then conducts data analysis and training on the health model through deep learning in the neural network. Then, the clipping treatment of cerebral aneurysm was analyzed, and finally, the treatment plan of clipping treatment of cerebral aneurysm based on the data analysis health model was designed. To verify the performance of the data analysis health model, this paper designs experiments on unbalanced data sets and experiments to improve the efficiency of algorithm execution. The data obtained through the experiment are analyzed, and then the data analysis health model is optimized, and finally, the clinical experiment is concluded. Compared with the traditional clipping treatment of cerebral aneurysm, the surgical success rate and postoperative recovery of the clipping treatment plan for cerebral aneurysm based on the data analysis health model designed in this paper are significantly improved.

The article "Clinical Treatment and Nursing Intervention Study of Clipping Treatment of Cerebral Aneurysm under the Health Model of Data Analysis" was retracted in 2023. Reasons: signs of a paper mill; suspected computer-generated content; unreliable results or conclusions; lack of ethics approval or compliance.

## Figures and Tables

**Figure 1:** Fields covered by big data.

**Figure 2:** The development process map of China's health and medical informatization.

**Figure 3:** Classification problem.

**Figure 4:** Flow chart of health big data classification.

**Figure 5:** Sketch of the neuron model.

**Figure 6:** Three-layer neural network model diagram.

**Figure 7:** Comparison of experimental results. (a). Comparison of classification accuracy results when cv = 10. (b). Comparison of ROC curve results.

**Figure 8:** Experimental results. (a). Comparison of detection of outliers by the algorithm before and after improvement. (b). Comparison of AUC changes of different algorithms.

**Figure 9:** Results of tumor observation experiment. (a). DSA measurement results. (b). 3D-DSA measurement results.

**Figure 10:** Comparison of results with traditional treatment regimens. (a). Surgical treatment success rate. (b). Degree of recovery after surgery.

**Table 1:** Detailed description of the three data sets.

Data set	Number of attributes	Number of samples	Minority class samples	Majority class samples	Nonequilibrium rate (%)
Glass	10	214	29	185	13.6
Adult	14	48842	12732	36110	26.1
Haberman	3	306	81	225	26.5

**Table 2:** Comparison of classification accuracy results.

Data set	Glass	Adult	Haberman
Original data set	0.6542	0.6669	0.6937
Traditional SMOTE processing	0.7319	0.7523	0.7875
Improved SMOTE handling	0.7748	0.7842	0.8273

**Table 3:** AUC area result comparison table.

Data set	Glass	Adult	Haberman
Original data set	0.6812	0.7043	0.7137
Traditional SMOTE processing	0.7511	0.7685	0.7963
Improved SMOTE handling	0.7885	0.7933	0.8273

**Table 4:** F1-Measure result comparison table.

Data set	Glass	Adult	Haberman
Original data set	0.7041	0.6829	0.7337
Traditional SMOTE processing	0.7897	0.8185	0.8212
Improved SMOTE handling	0.8159	0.8433	0.8533

**Table 5:** AUC area of different algorithms on different data sets.

Algorithm	Original data set	Outlier detection	Improve outlier detection
Tri-training	0.7692	0.8533	0.8704
K-means	0.7014	0.7473	0.7562
SVM	0.7852	0.8221	0.8312

## Data Availability

No data were used to support this study.
